The article "Deep Image Watermarking to JPEG Compression Based on Mixed-Frequency Channel Attention" was retracted in 2023. Reasons: unreliable results or conclusions; concerns about the data; concerns about the peer review; concerns about the citations.

# Deep Image Watermarking to JPEG Compression Based on Mixed-Frequency Channel Attention

**DOI:** 10.1155/2022/9880038

**Published:** 2022-07-14

**Authors:** Jun Tan, Yinan Hu, Ziming Shi, Bin Wang

**Affiliations:** ^1^The Key Laboratory of Advanced Design and Intelligent Computing, School of Software Engineering, Dalian University, Dalian 116622, China; ^2^Dalian University Experimental Center, Dalian University, Dalian 116622, China

## Abstract

Deep blind watermarking algorithms based on an end-to-end encoder-decoder architecture have recently been extensively studied as an important technology for protecting copyright. However, none of the existing algorithms can fully utilize the channel features of the image to improve the robustness against JPEG compression while obtaining high visual quality. Therefore, we propose firstly a mixed-frequency channel attention method in the encoder, which utilizes different frequency components of the 2D-DCT domain as weight coefficients during channel squeezing and excitation. Its essence is to suppress the useless feature maps and enhance the feature maps suitable for watermarking embedding by introducing frequency analysis in the channel dimension. The experimental results indicate that the PSNR of our method reaches over 38 and the BER is less than 0.01% under the JPEG compression with quality factor *Q* = 50. Besides, the proposed framework also obtains excellent robustness for a variety of common distortions, including Gaussian filter, crop, crop out, and drop out.

## 1. Introduction

As the mobile Internet industry develops rapidly, people gain access to large amounts of multimedia information. However, the deluge of multimedia information has resulted in a series of issues, including copyright conflicts and malicious tampering. Image encryption [1, 2], steganography [3, 4], digital watermarking [5], and other technologies came into being to solve the problem caused by information leakage. Digital watermarking, an effective technology for protecting copyright, has been used in image, audio, video, and other fields [6–11]. Digital image watermarking is one of the most important research directions for digital watermarking. The principle of digital image watermarking is to embed secret messages into the cover image in a way that is imperceptible to the human visual system, and the secret messages can still be recovered even if the encoded image is modified.

Traditional digital image watermarking algorithms are mainly divided into spatial watermarking and frequency watermarking. The spatial watermarking algorithms embed the watermark directly by modifying the image pixel, but this method is easily detected by a statistical method [12]. Therefore, researchers began to pay attention to the frequency domain, and they found that watermark embedding in DCT [13], DWT [14], and other frequency domains has better robustness and image visual quality. However, these traditional methods rely heavily on artificial shallow feature extraction, and they cannot make full use of the cover image, which greatly limits the robustness of the algorithm.

The article "Deep Image Watermarking to JPEG Compression Based on Mixed-Frequency Channel Attention" was retracted in 2023. Reasons: unreliable results or conclusions; concerns about the data; concerns about the peer review; concerns about the citations.

In recent years, with the success of deep neural networks in information hiding [15, 16] and other fields [17–21], some digital watermarking algorithms based on the deep neural network (DNN) have emerged [22, 23]. Kandi et al. [24] firstly applied a Convolutional Neural Network (CNN) to watermarking, which offers superior invisibility and robustness over traditional methods. However, the method is nonblind watermarking, which only applies in a narrow area. Ahmadi et al. [25] proposed a blind watermarking based on CNN, in which the circular convolution blocks are used to expand secret messages into the whole cover image to withstand geometric distortions. Zhu et al. [26] proposed an end-to-end DNN-based model for watermarking and a method called JPEG-Mask, which simulates the nondifferential JPEG compression. However, the simulated JPEG compression added as a noise layer to the training cannot achieve the effect that real JPEG compression plays. Therefore, a two-stage separable deep watermarking framework [27] was proposed. In stage I, only the encoder and decoder were initially trained to perform powerfully in encoding and decoding, and the decoder is individually fine-tuned by nondifferential distortions in stage II. The two-stage method may find the locally optimal results but cannot find the globally optimal results. Jia et al. [28] proposed a Mini-Batch of Real and Simulated JPEG compression (MBRS) method. For each minibatch image, one of the simulated JPEG, real JPEG compression, and a noise-free layer (identity) is selected randomly as the noise layer, and the gradient direction is updated in real time to find the globally optimal result. However, the above-mentioned methods ignore the frequency analysis, which can be combined with channel feature selection to improve the visual quality and robustness.

In order to address the aforementioned problems, based on the previous work [29, 30] about frequency analysis being introduced into DNN, we proposed a new attention method in this paper, which consists of two branches. One branch utilizes several squeeze-and-excitation (SE) [31] blocks to extract the lowest-frequency components of the DCT domain [32] from the channel feature maps to obtain the basic information of the cover image. The other branch utilizes frequency channel attention (FCA) [29] blocks to extract the low-frequency components of channel feature maps to reserve some details. Intuitively, we think that multifrequency components can capture more details to improve visual quality and the combined components of channels can withstand JPEG compression. Besides, we add a diffusion block that is a fully connected layer used in [28] into the message processor to diffuse the secret message into the whole image. In our architecture, we use the strength factor to adjust the trade-off between robustness and imperceptibility. The results indicate that under JPEG compression, our method can achieve higher image quality and the decoding bit error rate (BER) is close to almost 0%. Moreover, we can train a model with a combined noise layer, making it robust for many common distortions.

The article "Deep Image Watermarking to JPEG Compression Based on Mixed-Frequency Channel Attention" was retracted in 2023. Reasons: unreliable results or conclusions; concerns about the data; concerns about the peer review; concerns about the citations.

In summary, the contributions of this paper are as follows:

- To our knowledge, we are the first to introduce the frequency channel attention into digital watermarking, and we propose a mixed-frequency channel attention method for robust and blind image watermarking
- We choose 16 low-frequency channel components according to the zigzag form as the compression weight coefficients for the FCA channel attention block in our proposed scheme. Experimental results show that this selection scheme is superior to the midfrequency and high-frequency components when the noise layer is JPEG compression
- We propose a two-branch structure, which concentrates on the information from the lowest-frequency channel feature map and other low-frequency channel feature maps. The results of the experiments indicate that this structure can perform better than other mixed-frequency channel attention structures

The remainder of the paper is arranged as follows.  Section 2 introduces the details of the proposed framework. Experiments and comparisons with relative schemes are presented in Section 3. The discussion and analyses are described in Section 4.  Section 5 concludes the paper.

## 2. Proposed Framework and Method

### 2.1. Network Architecture

As shown in Figure 1, the whole model includes five components: message processor, encoder, noise layer, decoder, and adversary.

#### 2.1.1. Message Processor MP

The message processor is mainly responsible for processing the message and inputting the processed feature maps into the encoder. MP receives the binary secret message *M* of length *l* that is composed of {0, 1} and outputs the message feature maps *M*_en_ of shape *C*′ × *H* × *W*, where *C*′ is the channel number of the feature map. Specifically, the message *M* is generated randomly with a length of *l* and is reshaped to {0, 1}^1×*h*×*w*^. It is then amplified by a 3 × 3 ConvBNReLU layer, which consists of a convolutional layer, batch normalization, and ReLU activation function and is expanded to *C* × *H* × *W* by several transposed convolution layers. Finally, to expand the message more appropriately, the features of the message are extracted by several SE blocks that maintain the shape.

The article "Deep Image Watermarking to JPEG Compression Based on Mixed-Frequency Channel Attention" was retracted in 2023. Reasons: unreliable results or conclusions; concerns about the data; concerns about the peer review; concerns about the citations.

#### 2.1.2. Encoder *E*

An encoder with the parameter *θ*_*E*_ takes a RGB color image *I*_co_ of the shape 3 × *H* × *W* and the message maps *M*_en_ as input and outputs an encoded image *I*_en_ of the shape 3 × *H* × *W*. For selecting channel features better, we utilize a mixed-frequency channel attention block that includes several SE blocks and an FCA block as shown in Figure 1. The whole encoder consists of several 3 × 3 ConvBNReLU layers, a mixed-frequency channel attention block, and a 1 × 1 convolutional layer. Firstly, we amplify the cover image through a 3 × 3 ConvBNReLU layer and then extract image features of the same shape with the proposed attention block. The feature maps obtained by the attention block are then concentrated through a 3 × 3 ConvBNReLU layer. We feed the cover image features and message feature maps obtained from the message processor into a 3 × 3 ConvBNReLU layer for simple fusion. Then, we concatenate the obtained tensor and the cover image into a new tensor and feed it into a 1 × 1 convolutional layer to obtain the encoded image *I*_en_. Training the encoder is aimed at minimizing the *L*_2_ distance between *I*_co_ and *I*_en_ by updating *θ*_*E*_:

(1) $$\begin{array}{c} L_{E_{1}}=\text{MSE}\left(I_{\text{co}},I_{\text{en}}\right)=\text{MSE}\left(I_{\text{co}},E\left(\theta_{E},I_{\text{co}},M_{\text{en}}\right)\right). \end{array}$$

#### 2.1.3. Noise Layer *N*

The robustness of the whole model is provided by the noise layer. We select different noises from the appointed noise pool as the noise layer. It receives *I*_en_ and outputs the noised image *I*_no_ of the same shape. Besides, the end-to-end model requires all noises to join in the process of training. Therefore, we proposed the MBRS method [28] as the training method for the noise layer.

#### 2.1.4. Decoder *D*

The task of the decoder with parameter *θ*_*D*_ is to recover the secret message *M*_*D*_ of length *L* from the noised image *I*_no_. The component determines the ability of the whole model to extract watermarking. In the decoding stage, we feed the noised image *I*_no_ to a 3 × 3 ConvBNReLU layer and downsample the obtained feature maps by several SE blocks. Then, we convert the multichannel tensor into a single-channel tensor through a 3 × 3 convolutional layer and change the shape of the single-channel tensor to obtain the decoded message *M*_*D*_. The objective of decoder training is to minimize the distance between *M* and *M*_*D*_ by updating parameters *θ*_*D*_ to make them the same:

(2) $$\begin{array}{c} L_{D}=\text{MSE}\left(M,M_{D}\right)=\text{MSE}\left(M,D\left(\theta_{D},I_{\text{no}}\right)\right). \end{array}$$

Since it plays an important role in the bit error rate indicator, the loss function accounts for the largest proportion of the total loss function.

The article "Deep Image Watermarking to JPEG Compression Based on Mixed-Frequency Channel Attention" was retracted in 2023. Reasons: unreliable results or conclusions; concerns about the data; concerns about the peer review; concerns about the citations.

#### 2.1.5. Adversary Discriminator *A*

The adversary discriminator [33] consists of several 3 × 3 ConvBNReLU layers and a global average pooling layer. Under the influence of the adversarial network, the encoder will try to deceive the adversary as much as possible, so that the adversary cannot make a correct judgment on *I*_co_ and *I*_en_. And update parameters *θ*_*E*_ to minimize *L*_*E*_2__ to improve the encoding visual quality of the encoder:

(3) $$\begin{array}{c} L_{E_{2}}=\log\left(A\left(\theta_{A},I_{\text{en}}\right)\right)=\log\left(A\left(\theta_{A},E\left(\theta_{E},I_{\text{co}},M_{\text{en}}\right)\right)\right). \end{array}$$

The discriminator with parameters *θ*_*A*_ needs to distinguish between *I*_co_ and *I*_en_ as a binary classifier. The goal of the adversary is to minimize the loss of classification *L*_*A*_ by updating *θ*_*A*_:

(4) $$\begin{array}{c} L_{A}=\log\left(1-A\left(\theta_{A},E\left(\theta_{E},I_{\text{co}},M_{\text{en}}\right)\right)\right)+\log\left(A\left(\theta_{A},I_{\text{co}}\right)\right). \end{array}$$

The total loss function is *L* = *λ*_*E*_*L*_*E*_1__ + *λ*_*D*_*L*_*D*_ + *λ*_*A*_*L*_*E*_2__, and loss *L*_*A*_ is for the adversary discriminator.

### 2.2. Squeeze-and-Excitation Networks

An SE channel attention mechanism focuses on exploring the correlation of channel dimensions by modelling the relationships between channels and adaptively adjusting the feature values of each channel so that the attention network learns global information and reinforces the useful information while suppressing the useless information. The SE channel attention network is divided into two-step operations including squeeze and excitation. Squeeze is specifically a global average pooling operation that compresses the size of feature map from *C* × *h* × *w* into *C* × 1 × 1, the result of which can represent global information. The excitation operation can be considered a combination of two fully connected layers. The tensor obtained after the squeeze operation is first fully connected to compress the *C* dimensional tensor to *C*/*r* dimension and activated by the ReLU function and then fully connected again to transform the *C*/*r* dimension back to *c* dimension and activated by the sigmoid function to obtain the weight tensor. Finally, the weight tensor with 1 × 1 obtained by the excitation operation is scaled by the original tensor with *C* × *h* × *w*.

The article "Deep Image Watermarking to JPEG Compression Based on Mixed-Frequency Channel Attention" was retracted in 2023. Reasons: unreliable results or conclusions; concerns about the data; concerns about the peer review; concerns about the citations.

### 2.3. Frequency Channel Attention

#### 2.3.1. The Basic Principle on FCA

Previous studies have tried to explain the relationship between the DCT and global average pooling (GAP) and hoped to mine the information of the DCT domain to better extract features from channels. In this section, we firstly review the formulas of 2D-DCT and GAP, and then, based on the aforementioned work, we elaborate on the principle of the FCA block and the selection of frequency components.

To express the basic functions of the two-dimensional (2D) DCT and the entire 2D-DCT more simply, we removed some constant normalization coefficients, but they did not affect the results, just a principle explanation:

(5) $$\begin{array}{c} b_{u,v}^{i,j}=\cos\left(\frac{\pi u}{H}\left(i+\frac{1}{2}\right)\right)\cos\left(\frac{\pi v}{W}\left(j+\frac{1}{2}\right)\right), \end{array}$$

(6) $$\begin{array}{c} F_{u,v}^{2d}=\overset{H-1}{\underset{i=0}{\sum }}\;\overset{W-1}{\underset{j=0}{\sum }}\;x_{i,j}^{2d}b_{u,v}^{i,j}. \end{array}$$

*F* ^2*d*^ is the computed 2D-DCT transform domain matrix, *x*^2*d*^ is the input, *H* is the height of *x*^2*d*^, *W* is the width of *x*^2*d*^, and *u* ∈ {0, 1, ⋯, *H* − 1} and *v* ∈ {0, 1, ⋯, *W* − 1}. GAP is a special case of 2D-DCT when *u* = 0 and *v* = 0 in equation (6), and its result is proportional to the lowest-frequency component of 2D-DCT and is confirmed in [29]:

(7) $$\begin{array}{c} F0,0^{2d}=\overset{H-1}{\underset{i=0}{\sum }}\;\overset{W-1}{\underset{j=0}{\sum }}\;x_{i,j}^{2d}\cos\left(\frac{0}{H}\left(i+\frac{1}{2}\right)\right)\cos\left(\frac{0}{W}\left(j+\frac{1}{2}\right)\right)=\text{gap}\left(x^{2d}\right)HW. \end{array}$$

The input to the channel attention block is divided into many parts along the channel dimension. A corresponding 2D-DCT frequency component is assigned to each part, and the 2D-DCT-transformed results can be used as the compression results of channel attention. All transformed parts are concatenated to produce a complete compressed vector. Finally, the obtained compressed weight tensor with 1 × 1 × *C* and the original input tensor are multiplied to get the final result.

### 2.4. Criteria for Choosing Frequency Components

According to the above proof, the squeezing operation of the SE attention block is equivalent to the lowest-frequency component in the corresponding 2D-DCT coefficients. Usually, this component concentrates on most of the energy information of the image, and the conclusion is also valid for channel features. SEnets are a very effective attention network used in most computer vision tasks, but most of the frequency domain components are discarded, some of which are beneficial to improve the performance of watermarking and should not be excluded. Therefore, in order to better compress the channel and introduce more information, we used the FCA block to expand the GAP to more 2D-DCT frequency components. Specific details of the implementation are shown in Figure 2(a). We divide 8 × 8 blocks according to the principle of JPEG compression and select the lowest-frequency component and 15 other low-frequency components according to the form of zigzag as the coefficients of the squeezing operation in the FCA block, as shown in Figure 2(b).

The article "Deep Image Watermarking to JPEG Compression Based on Mixed-Frequency Channel Attention" was retracted in 2023. Reasons: unreliable results or conclusions; concerns about the data; concerns about the peer review; concerns about the citations.

### 2.5. Noise Layer

#### 2.5.1. JPEG Compression

In the real JPEG compression process, we need to quantize the DCT coefficients according to the quantization tables and round them up to the nearest whole number, but the process is nondifferential, which means that the gradient propagates back and the decoding loss will be zero. To address the above-mentioned problem, we use the MBRS method, which can effectively solve the problem about nondifferential distortions.

#### 2.5.2. Traditional Noise Attack

In the field of blind watermarking, some typical noises are often used to test the robustness of the model. In our work, we train five different models separately on the noises, which include crop (*p* = 0.035), crop out (*p* = 0.3), drop out (*p* = 0.3), Gaussian filter (*σ* = 2), and identity. Besides, we train a combined noise model with JPEG-Mask (*Q* = 50), JPEG (*Q* = 50), crop (*p* = 0.0225), and identity, which can resist most of the distortions.

### 2.6. Strength Factor

We use *I*_diff_ = *I*_en_ − *I*_co_ to represent the residual signal between the encoded image and the cover image and adjust the trade-off between the visual quality and the bit error rate by the strength factor *S*: *I*_en,*s*_ = *I*_co_ + *S* · *I*_diff_. The generated image *I*_en,*s*_ is fed into the noise layer to obtain the noised image *I*_no_. We keep *S* on 1 in the training process and change the *S* in the testing process for different applications. Because our method is a blind watermarking, the trick is used only in the encoder.

## 3. Experiments and Results

### 3.1. Experimental Setup, Metrics, and Baselines

To evaluate the effectiveness of the proposed method, we use 10000 random images from the ImageNet dataset [34] for training and 5000 images from the COCO dataset [35] for testing, aiming at ensuring the generation of the trained model. We select the JPEG compression function in the PIL package as testing. The strength factor is set as 1 during training. For the weight factors of the loss function, we choose *λ*_*E*_ = 1, *λ*_*D*_ = 10, and *λ*_*A*_ = 0.0001. For the optimized function, Adam [36] is applied with a learning rate of 10^−3^ and default hyperparameters. Each model is trained for 100 epochs with a batchsize 16. PSNR and SSIM [37] measure the similarity between *I*_en_ and *I*_co_. Robustness is measured by the the difference called BER between the decoded message and secret message. Our baselines for comparison are [26, 27] and [28]. In pursuit of the real results, we realize the MBRS [28] based on the open source of both codes and models. We also try to conduct experiments of [26, 27] but could not reproduce the best performance that they reported. In order to respect the results that they reported, we directly use their published results.

The article "Deep Image Watermarking to JPEG Compression Based on Mixed-Frequency Channel Attention" was retracted in 2023. Reasons: unreliable results or conclusions; concerns about the data; concerns about the peer review; concerns about the citations.

### 3.2. Comparison with SOTA Methods

#### 3.2.1. Robustness

We train a model with JPEG-Mask (*Q* = 50), real JPEG (*Q* = 50), and identity to demonstrate the robustness of our model against JPEG compression. All the testing processes are performed under real JPEG (*Q* = 50). As shown in Table 1, compared to the other method, our model achieves the PSNR that is higher than 38 and the BER that is less than 0.01%, which indicates that our model not only maintains higher image quality for JPEG compression but also achieves lower BER.  Figure 3 indicates that the messages are embedded in most areas of the cover images. In addition to JPEG compression distortion, our model is also robust to other image processing distortions, such as Gaussian filter (GF), crop, crop out, and drop out. We also train a combined noise model to embed a 30-bit message into 128 × 128 images with the noise layer consisting of JPEG-Mask (*Q* = 50), real JPEG (*Q* = 50), identity, and crop (*p* = 0.0225) and add a diffusion and an inverse-diffusion block mentioned in [28] into the message processor for diffusing a secret message to the whole cover image to resist geometry attacks. As shown in Table 2, our trained model shows robustness against most noises. We also tested some noises not included in the noise layer for the combined noise model, and the experimental results are shown in Figure 4.

#### 3.2.2. Transparency

In order to show that our method can learn more frequency features from cover images, we separately train five models with the noise layer. For GF (*σ* = 2) and identity, we embed 64-bit messages into 3 × 128 × 128 images without a diffusion block. For crop (*p* = 0.035), crop out (*p* = 0.3), and drop out (*p* = 0.3), we embed 30-bit messages into 3 × 128 × 128 images with the diffusion block. Besides, we compare the PSNR and SSIM between *I*_co_ and *I*_en_ by adjusting *S* under roughly the same BER. As shown in Table 3, the results of the proposed method perform better than those of other models under most distortions, but our specialized trained model performs worse for the crop attack. Since the information diffusion block we use has more information embedded on a single channel, it has some shortcomings compared to [26] of broadcasting single-bit information on a single channel.

The article "Deep Image Watermarking to JPEG Compression Based on Mixed-Frequency Channel Attention" was retracted in 2023. Reasons: unreliable results or conclusions; concerns about the data; concerns about the peer review; concerns about the citations.

### 3.3. Ablation Study

#### 3.3.1. Strength Factor

The strength factor is a parameter used to balance robustness and imperceptibility. We set the value of the strength factor *S*, from 0.1 to 2.0, with an interval of 0.1, and test the model under different quality factors for JPEG compression. The results are shown in Table 4. With the increment of *S*, PSNR and SSIM values decrease, the quality of the encoded image becomes worse, and the extraction accuracy becomes higher. In the study, we adjust the value of *S* to obtain the similar visual quality of different models for fair comparison.

#### 3.3.2. Discriminator

To demonstrate that the discriminator can help the encoder generate higher-quality images, we trained the noise-free model with and without the discriminator separately. As can be seen from the normalized watermarking residuals in Figure 5, the watermarking model without the discriminator does not produce a uniform distribution of watermarking and produces visual artifacts on the resulting watermarked image. However, the watermarking model with a discriminator generates an even distribution of watermarking, and no aggregation of watermarking occurs.

#### 3.3.3. Different Mixed-Frequency Channel Attention

To demonstrate that our two-branch structure is superior to other combined mixed-frequency channel attention blocks, we conduct experiments for the encoder with different frequency channel attention structures. We proposed another four kinds of structures to be applied in the encoder. The first is called LFCA, which only consists of several FCA blocks with low-frequency components, the second is called SE&LFCA, in which we insert an FCA block behind the SE blocks, the third is composed of several SE blocks, and the last is called LFCA&SE, in which we insert an FCA block in front of the SE blocks. Their detailed structures are shown in Figure 6. We list the results of experiments separately under JPEG compression and combined noises for the above-mentioned four structures in Tables 5 and 6.

The channel attention mechanism assigns weights to the feature maps. SE only selects the lowest-frequency component coefficients of the 2D-DCT to enhance all channel feature maps through multiple SE blocks, while LFCA chooses to divide the feature maps on the channels and select multiple low-frequency component coefficients of the 2D-DCT to enhance through several LFCA blocks. We believe that when the noise layer only includes JPEG compression, the weights of LFCA enhancement are spread over multiple low-frequency components relative to SE, and thus, the performance will be worse than that of SE. However, combining SE blocks and LFCA blocks gives better performance. As can be seen from Table 5, the performance of SE&LFCA and LFCA&SE is better than that of SE and LFCA. SE&LFCA firstly allocates the lowest-frequency component coefficients through an SE block and then uses several LFCA blocks to enhance multifrequency component coefficients on the basis of the lowest-frequency component, which has a good effect. Although LFCA&SE is also composed of an SE block and several LFCA blocks, its effect is not as good as that of SE&LFCA. We believed that this is caused by LFCA assigning weights in the first place.

The article "Deep Image Watermarking to JPEG Compression Based on Mixed-Frequency Channel Attention" was retracted in 2023. Reasons: unreliable results or conclusions; concerns about the data; concerns about the peer review; concerns about the citations.

Our parallel structure is a better way of feature fusion when the noise layer includes multinoises. We believe that the reason why the experimental results of SE&LFCA and LFCA&SE perform worse is that they have no skip connection. Our proposed method achieves better performance with skip connection of FCA, which is confirmed by the experimental results in Table 7.

#### 3.3.4. Selection Scheme of Frequency Components

To demonstrate that the FCA attention block in our method chooses the low-frequency component coefficients of the DCT to improve the robustness to JPEG compression, we select 16 components of low frequency, 16 components of middle frequency, and 16 components of high frequency as the weight coefficients of FCA from the 8 × 8 coefficients, respectively, and train them under JPEG compression. It can be seen from Table 8 that the selection of frequency domain components has a certain impact on the robustness and imperceptibility of the model. When the low-frequency components are selected, the metrics such as PSNR, SSIM, and BER all reach the highest.

#### 3.3.5. Skip Connection

To show the important role of introducing frequency analysis and skip connection, we trained three different watermarking models under a mixed-noise layer separately: baseline: without attention networks in the encoder; +SE: with the addition of the SE channel attention blocks in the encoder; and +skip connection: based on +SE, with the addition of the LFCA attention block via skip connection. Table 7 shows the results of experiments, where the performance of the model by adding SE attention block is improved compared to baseline under most of the noises. However, we find that the embedding of the watermark information by adding the SE attention block is more concentrated in the low-frequency region which is less affected by the Gaussian filter but will be more affected by the Gaussian noise. In order to further improve the robustness for noises such as JPEG compression, we added the LFCA attention block by skip connection on the basis of the SE attention blocks, and the experimental results show that the quality of the encoded image is improved by skip connection, the best robustness is achieved for most distortions, and our watermark embedding assignment is more reasonable.

The article "Deep Image Watermarking to JPEG Compression Based on Mixed-Frequency Channel Attention" was retracted in 2023. Reasons: unreliable results or conclusions; concerns about the data; concerns about the peer review; concerns about the citations.

## 4. Discussion and Analysis

According to Figures 2, 3, and 6 and Tables 5 and 6, some analyses are given as follows.

1. Our scheme significantly improved visual quality compared with relative schemes. We can find that the secret messages are embedded in most areas of the cover image including low-frequency and high-frequency components from Figure 3
2. To further reflect our scheme, we calculated the indicators SSIM and PSNR. SSIM can show the overall structure of images. PSNR is calculated based on the discrepancy between the corresponding two pixel values. PSNR and SSIM are utilized jointly to evaluate the visual quality of the encoded image
3. A frequency channel attention block with selected low-frequency channel components can effectively improve the robustness and imperceptibility of the proposed watermarking model under JPEG compression and combined noise layer, as shown in Tables 5 and 6. However, the performance of the variants suggests that the balance of robustness and invisibility is very challenging. Our scheme chose the two-branch structure to concentrate on the features from the LFCA block and SE blocks. Experimental results demonstrate that skip connections provide better performance gains for the whole model
4. The performance of the watermarking algorithm depends largely on the selection of frequency channel components. We chose 16 low-frequency channel components according to the zigzag form. Compared to the lowest-frequency channel components extracted by the SE block and medium-high-frequency channel components, the multi-low-frequency channel components include the information that is beneficial to embedding messages and defence distortions
5. Although the method we proposed at the current stage has good performance in robustness and imperceptibility, we believe that it will also cause computational costs to a certain extent. Therefore, we hope to explore more concise and effective selection methods of channel feature components in the future

The article "Deep Image Watermarking to JPEG Compression Based on Mixed-Frequency Channel Attention" was retracted in 2023. Reasons: unreliable results or conclusions; concerns about the data; concerns about the peer review; concerns about the citations.

## 5. Conclusions

In the paper, we proposed a novel mixed-frequency channel attention block to improve the robustness and imperceptibility of existing deep robust image watermarking algorithms for JPEG compression. We divide the 2D-DCT frequency space into 8 × 8 parts according the principle of JPEG compression and utilize the SE block to obtain the lowest-frequency component in 2D-DCT domain, which is equal to GAP operation, as the weight coefficient for input. Then, we select the 16 low-frequency components in the 2D-DCT domain as the weight coefficients by the FCA block according to the zigzag form. Finally, we concentrate on the feature maps by skip connection in the channel dimension. Besides, we use an optional diffusion block in [28] for robustness against geometric attack. The comprehensive experiments have proven that the proposed method performs better in not only robustness but also image quality. Skip connection and the selection scheme of frequency components prove to be effective. In the future, we will also explore a more suitable channel selection method for watermarking embedding.

## Figures and Tables

**Figure 1:** Overall model architecture. The message processor can learn the method for expanding message and realizing redundancy by the transposed convolutional layer; the encoder includes the mixed-frequency channel attention block which embeds the secret message into the whole cover image, the noise layer changes the kind of noise according to the MBRS method for offering the robustness, and the decoder extracts the secret message from the encoded image. An adversary discriminator is used to distinguish the cover image and the encoded image.

**Figure 2:** (a) The working theory of the FCA block. (b) The method of selecting frequency components in the DCT domain.

**Figure 3:** Examples of showing the robustness of the model against JPEG compression (*Q* = 50) with experimental results. From top to bottom are the cover images, the encoded images, the noised images, the residual between cover images and encoded image, and the normalization of the residual signal.

**Figure 4:** Robustness against different traditional noises. We tested different noises including those that were not included in the trained combined noise layer under strength factor *s* = 1. The combined noise layer consists of JPEG-Mask (*Q* = 50), real JPEG (*Q* = 50), identity, and crop (*p* = 0.0225). Top: cover image *I*_co_; second: encoded image *I*_en_; third: noised image *I*_no_; fourth: residual between *I*_no_ and *I*_co_; and bottom: the normalization of the residual signal.

**Figure 5:** The results of encoding with and without a discriminator: top: cover image *I*_co_; second: encoded image *I*_en_; third: noised image *I*_no_; fourth: residual signal between *I*_en_ and *I*_co_; and bottom: the normalization of the residual signal.

The article "Deep Image Watermarking to JPEG Compression Based on Mixed-Frequency Channel Attention" was retracted in 2023. Reasons: unreliable results or conclusions; concerns about the data; concerns about the peer review; concerns about the citations.

**Figure 6:** The other structures of mixed-frequency channel attention, which are proposed in the ablation experiment. The structure called LFCA is only composed of several frequency channel attention blocks with low-frequency components. The structure called SE consists of several SE channel attention blocks. The structure called SE&LFCA inserts an FCA block behind the SE blocks. The structure called LFCA&SE inserts FCA blocks in front of the SE blocks.

**Table 1:** Comparison with the SOTA. We realized the model opening source in [28], while directly using the results included as reported in [26, 27] under quality factor 50. However, SSIM is not reported in [26, 27], for which we empty these items. PSNR is measured for RGB channels, except in [26]; they use the Y channel of the YUV color space.

Model	HiDDeN [26]	TSDL [27]	MBRS [28]	Ours
Image size	128 × 128	128 × 128	128 × 128	128 × 128
Message length	30	30	64	64
Noise layer	JPEG-Mask	JPEG	Mixed	Mixed
PSNR	30.09	33.51	36.49	38.13
SSIM	—	—	0.9173	0.9472
BER	15%	22.3%	0.0092%	0.0078%

**Table 2:** Results of robustness against other distortions. We add an additive diffusion block into the message processor for improving the shortcoming that our original structure is not robust enough against crop, crop out, and drop out and make a comparison with [26–28] trained by a combined noise layer. The strength factor is adjusted for comparison under PSNR = 33.5.

Noise	Identity	Crop out (*p* = 0.3)	Drop out (*p* = 0.3)	Crop (*p* = 0.035)	GF (*σ* = 2)	JPEG (*Q* = 50)
HiDDeN [26]	0%	6%	7%	12%	4%	37%
TSDL [27]	0%	2.7%	2.6%	11%	1.4%	23.8%
MBRS [28]	0%	0.0027%	0.0087%	4.15%	0.011%	4.48%
Ours	0%	0.0013%	0.0080%	3.24%	0.293%	2.61%

**Table 3:** Results of transparency against other distortions. For revealing the advantage of our proposed method, we make a comparison of PSNR and SSIM with [26, 28] by adjusting strength factor *S* to keep the BER at 0%. Because the experiment of [27] is not done, we do not list it.

Metric	Model	Crop (*p* = 0.035)	Crop out (*p* = 0.3)	Drop out (*p* = 0.3)	GF (*σ* = 2)	Identity
PSNR	HiDDeN [26]	35.20	47.24	42.52	40.55	44.63
	MBRS [28]	32.15	46.77	48.50	40.74	42.81
	Ours	33.01	47.26	49.43	42.30	45.71

SSIM	HiDDeN [26]	—	—	—	—	—
	MBRS [28]	0.7872	0.9910	0.9936	0.9670	0.9740
	Ours	0.8225	0.9924	0.9945	0.9760	0.9867

BER	HiDDeN [26]	0%	3%	0%	0%	0%
	MBRS [28]	0.72%	0%	0%	0%	0%
	Ours	0.29%	0%	0%	0%	0%

**Table 4:** BER, PSNR, and SSIM values under different strength factors *S* and quality factors of JPEG *Q*.

Strength factor		0.4	0.6	0.8	1.0	1.2	1.4
BER	*Q* = 10	35.03%	27.91%	21.80%	16.86%	13.02%	10.06%
	*Q* = 30	15.65%	5.94%	1.63%	0.33%	0.047%	0.0053%
	*Q* = 50	7.74%	1.11%	0.0778%	0.0050%	0.0012%	0.00%
	*Q* = 70	3.87%	0.370%	0.0170%	0.0009%	0.00%	0.00%
	*Q* = 90	2.53%	0.202%	0.0078%	0.0006%	0.00%	0.00%

PSNR		45.92	42.40	39.89	37.95	36.37	35.03
SSIM		0.9893	0.9773	0.9623	0.9455	0.9274	0.9086

The article "Deep Image Watermarking to JPEG Compression Based on Mixed-Frequency Channel Attention" was retracted in 2023. Reasons: unreliable results or conclusions; concerns about the data; concerns about the peer review; concerns about the citations.

**Table 5:** Comparison with the ablation experimental results, with the best results in bold and second bests in blue. We compared the performance with four mixed-frequency channel attention variants under JPEG compression (*Q* = 50).

Model	SE	LFCA	SE&LFCA	LFCA&SE	Ours
Image size	128 × 128	128 × 128	128 × 128	128 × 128	128 × 128
Message length	64	64	64	64	64
Noise layer	Mixed	Mixed	Mixed	Mixed	Mixed
PSNR	37.70	37.32	**38.21**	37.49	38.13
SSIM	0.9445	0.9428	**0.9553**	0.9487	0.9472
BER	0.0082%	0.0081%	**0.0059%**	0.0081%	0.0078%

**Table 6:** BER comparison between the proposed scheme and ablation schemes, with the best results in bold, second bests in blue, and the worst results in red. The strength factor is adjusted for comparison under PSNR = 33.5.

Noise	Identity	Crop out (*p* = 0.3)	Drop out (*p* = 0.3)	Crop (*p* = 0.035)	GF (*σ* = 2)	JPEG (*Q* = 50)
SE	0%	0.0027%	0.0093%	5.07%	0.011%	3.22%
LFCA	0%	**0.0%**	**0.0027%**	4.23%	0.031%	5.62%
SE&LFCA	0%	0.0040%	0.0179%	6.21%	0.185%	22.87%
LFCA&SE	0%	0.0047%	0.0053%	18.06%	**0.006%**	9.12%
Ours	0%	0.0013%	0.0080%	**3.24%**	0.293%	**2.61%**

**(a):** 

Model	Metric	JPEG (*Q* = 50)	Crop (*p* = 0.035)	Crop out (*p* = 0.3)	Drop out (*p* = 0.3)	GF (*σ* = 2)
Baseline	PSNR	32.60	32.60	32.59	32.57	32.59
+SE		32.55	32.58	32.57	32.56	32.56
+skip connection (LFCA)		32.75	32.76	32.76	32.73	32.76

Baseline	SSIM	0.8150	0.8157	0.8149	0.8146	0.8150
+SE		0.8161	0.8165	0.8160	0.8157	0.8159
+skip connection (LFCA)		0.8263	0.8266	0.8263	0.8259	0.8265

Baseline	BER	3.09%	6.96%	0%	0.0007%	0.168%
+SE		2.19%	4.30%	0.0013%	0.0067%	0.0054%
+skip connection (LFCA)		1.94%	3.08%	0.0067%	0.0040%	0.228%

**(b):** 

Salt&Pepper (*p* = 0.1)	GN (*p* = 0.1)	MF (*s* = 3)
32.59	32.59	32.58
32.55	32.56	32.55
32.75	32.76	32.75

0.8148	0.8153	0.8154
0.8156	0.8159	0.8160
0.8260	0.8271	0.8263

0.830%	1.23%	0%
0.813%	1.51%	0%
0.665%	0.859%	0%

**Table 8:** BER comparison between the proposed scheme and ablation schemes. We train three different ways of frequency domain component selection for the FCA attention block in the mixed-frequency channel attention block under JPEG compression. Low frequency: 16 coefficients of low-frequency components; middle frequency: 16 coefficients of middle-frequency components; and high frequency: 16 coefficients of high-frequency components.

Model	PSNR	SSIM	BER
High frequency	37.77	0.9407	0.6781%
Middle frequency	38.02	0.9472	0.5782%
Low frequency	38.13	0.9472	0.0078%

The article "Deep Image Watermarking to JPEG Compression Based on Mixed-Frequency Channel Attention" was retracted in 2023. Reasons: unreliable results or conclusions; concerns about the data; concerns about the peer review; concerns about the citations.

## Data Availability

The dataset of this article was obtained from the dataset published on http://images.cocodataset.org/zips/train2014.zip and http://image-net.org/download.php.

## References

[1] Shi Y., Yinan H., Wang B. (2021). Image encryption scheme based on multiscale block compressed sensing and Markov model. *Entropy*.

[2] Zhou S. (2021). A real-time one-time pad DNA-chaos image encryption algorithm based on multiple keys. *Optics & Laser Technology*.

[3] Liao X., Yin J., Chen M., Qin Z. (2020). Adaptive payload distribution in multiple images steganography based on image texture features. *IEEE Transactions on Dependable and Secure Computing*.

[4] Xiaotian W., Yang C.-N. (2019). Partial reversible AMBTC-based secret image sharing with steganography. *Digital Signal Processing*.

[5] Xiong L., Han X., Yang C.-N., Shi Y.-Q. (2022). Robust reversible watermarking in encrypted image with secure multi-party based on lightweight cryptography. *IEEE Transactions on Circuits and Systems for Video Technology*.

[6] Bamatraf A., Ibrahim R., Mohd Najib B., Salleh M. Digital watermarking algorithm using LSB.

[7] Tao B., Dickinson B. Adaptive watermarking in the DCT domain.

[8] Barni M., Bartolini F., Cappellini V., Piva A. (1998). A DCT-domain system for robust image watermarking. *Signal Processing*.

[9] Swanson M. D., Zhu B., Tewfik A. H. (1998). Multiresolution scene-based video watermarking using perceptual models. *IEEE Journal on Selected Areas in Communications*.

[10] Bassia P., Pitas I., Nikolaidis N. (2001). Robust audio watermarking in the time domain. *IEEE Transactions on Multimedia*.

[11] Uchida Y., Nagai Y., Sakazawa S., Satoh S. I. Embedding watermarks into deep neural networks.

[12] Dumitrescu S., Wu X., Wang Z. (2003). Detection of LSB steganography via sample pair analysis. *International Workshop on Information Hiding*.

[13] Jiansheng M., Sukang L., Xiaomei T. (2009). A digital watermarking algorithm based on DCT and DWT.

[14] Shen Y., Tang C., Min X., Chen M., Lei Z. (2021). A DWT-SVD based adaptive color multi-watermarking scheme for copyright protection using AMEF and PSO-GWO. *Expert Systems with Applications*.

[15] Baluja S. (2020). Hiding images within images. *IEEE Transactions on Pattern Analysis and Machine Intelligence*.

[16] Jing J., Deng X., Mai X., Wang J., Guan Z. Hinet: deep image hiding by invertible network.

[17] Changqian Y., Wang J., Peng C., Gao C., Yu G., Sang N. Bisenet: bilateral segmentation network for real-time semantic segmentation.

The article "Deep Image Watermarking to JPEG Compression Based on Mixed-Frequency Channel Attention" was retracted in 2023. Reasons: unreliable results or conclusions; concerns about the data; concerns about the peer review; concerns about the citations.

[18] Isola P., Zhu J.-Y., Zhou T., Efros A. A. Image-to-image translation with conditional adversarial networks.

[19] Zhu J.-Y., Park T., Isola P., Efros A. A. Unpaired image-to-image translation using cycle-consistent adversarial networks.

[20] Song T., Zhang X., Ding M., Rodriguez-Paton A., Wang S., Wang G. (2022). DeepFusion: a deep learning based multi-scale feature fusion method for predicting drug-target interactions. *Methods*.

[21] Meng X., Li X., Wang X. (2021). A computationally virtual histological staining method to ovarian cancer tissue by deep generative adversarial networks. *Computational and Mathematical Methods in Medicine*.

[22] Plata M., Syga P. Robust spatial-spread deep neural image watermarking.

[23] Jamali M., Karim N., Khadivi P., Shirani S., Samavi S. (2021). Robust watermarking using diffusion of logo into autoencoder feature maps. https://arxiv.org/abs/2105.11095.

[24] Kandi H., Mishra D., Gorthi S. R. (2017). Exploring the learning capabilities of convolutional neural networks for robust image watermarking. *Computers & Security*.

[25] Ahmadi M., Norouzi A., Karimi N., Samavi S., Emami A. (2020). ReDMark: framework for residual diffusion watermarking based on deep networks. *Expert Systems with Applications*.

[26] Zhu J., Kaplan R., Johnson J., Fei-Fei L. HiDDeN: hiding data with deep networks.

[27] Liu Y., Guo M., Zhang J., Zhu Y., Xie X. A novel two-stage separable deep learning framework for practical blind watermarking.

[28] Jia Z., Fang H., Zhang W. MBRS: enhancing robustness of DNN-based watermarking by Mini-Batch of Real and Simulated JPEG compression.

[29] Qin Z., Zhang P., Fei W., Li X. Fcanet: frequency channel attention networks.

[30] Ehrlich M., Davis L. S. Deep residual learning in the JPEG transform domain.

[31] Jie H., Shen L., Sun G. Squeeze-and-excitation networks.

[32] Ahmed N., Natarajan T., Rao K. R. (1974). Discrete cosine transform. *IEEE Transactions on Computers*.

[33] Goodfellow I., Pouget-Abadie J., Mirza M. (2014). Generative adversarial nets. *Advances in Neural Information Processing Systems*.

[34] Deng J., Dong W., Socher R., Li L.-J., Li K., Fei-Fei L. ImageNet: a large-scale hierarchical image database.

[35] Lin T. Y., Maire M., Belongie S. Microsoft coco: common objects in context.

[36] Kingma D. P., Lei Ba J. Adam: a method for stochastic optimization.

[37] Hore A., Ziou D. Image quality metrics: PSNR vs. SSIM.

